# LSR Promotes Cell Proliferation and Invasion in Lung Cancer

**DOI:** 10.1155/2021/6651907

**Published:** 2021-03-08

**Authors:** Min Zhang, Cui Ma

**Affiliations:** ^1^Department of Respiratory Medicine, The Second Affiliated Hospital of Zhejiang University School of Medicine, 88 Jiefang Road, 310009 Hangzhou, Zhejiang, China; ^2^Department of Endocrinology, Zhejiang Greentown Cardiovascular Hospital, 409 Gudun Road, 310012 Hangzhou, Zhejiang, China

## Abstract

The lipolysis-stimulated lipoprotein receptor (LSR) displays an important regulatory role in cancer. However, the association between LSR and lung cancer is still elusive. Here, the candidate oncogene LSR on Ch.9q was obtained and assessed by bioinformatics analysis of The Cancer Genome Atlas (TCGA) dataset of lung cancer. We conducted clinical pathology and survival analysis based on the lung cancer database. We assessed the biological effects of LSR in lung cancer cells on cell proliferation. Our data indicated that LSR was upregulated in lung cancer cells. Meanwhile, LSR was identified in this study to be a poor prognostic factor, and its high expression exhibited relations with grades, stages, and nodal metastasis status. Using *in vitro* analysis, our data revealed that LSR could promote lung cancer progression by regulating cell proliferation, migration, and invasion. In our study, our data demonstrated that LSR was a tumor promoter for lung cancer and was a potential biomarker and target for lung cancer prognosis and treatment.

## 1. Background

Presently, lung cancer is becoming the pivotal inducer of male and female mortality worldwide. The global diagnosis rate of newly generated cases is about 1.6 million per year [1]. The poor prognosis may be due to the high proportion of advanced patients and the lack of active anticancer treatment for most early patients [2]. The probable reason for the high mortality of lung cancer is caused by genetic and environmental factors and tumor treatment [3]. The therapeutic efficacy of patients with lung cancer has been dramatically ameliorated after combined use of surgery, radiotherapy, and systemic therapy on patients with early disease [4]. Meanwhile, with the in-depth research on the molecular mechanism of lung cancer, the introduction of targeted therapies, immune methods, and chemotherapy in the treatment process has greatly improved the treatment methods for patients with advanced lung cancer [5]. However, it is still necessary to further explore reliable lung cancer phenotype markers to improve the effect of lung cancer treatment.

The locus of lipolysis-stimulated lipoprotein receptors (LSR) is at the upstream of apolipoprotein (Apo) E [6], which is a key risk factor for cardiovascular disease (CVD) [7]. LSR includes ApoB and ApoE receptors that participate in removing triglyceride-rich lipoproteins in the postprandial phase [8]. Since the common polymorphisms of ApoE can significantly affect the variability of lipid metabolism, LSR may be involved in the pathology of type III hyperlipidemia and cardiovascular disease [9]. LSR is the key molecule of the three-cell contact in the normal cell epithelial barrier and cancer cell malignancies [10]. In endometrial cancer and human pancreatic cancer, it has been found that the loss of LSR can induce the migration, invasion, and proliferation of cancer cells [11]. At the same time, LSR can damage the invasive properties of bladder cancer cells [12]. LSR can bind to lipoproteins rich in triglycerides and act as a lipoprotein receptor associated with certain malignant tumors [13]. LSR exhibits importance in gastric cancer development, indicating that it is a probable target in lung cancer therapy in the following study.

In this study, by searching in TCGA database, it was found that LSR might be a gene associated with lung cancer. We analyzed the correlation between the expression of LSR and the clinical parameters and prognostic value of lung cancer patients. Besides, the expression level of LSR affected the proliferation and metastasis of lung cancer cells.

## 2. Materials and Methods

### 2.1. Public Datasets

TCGA dataset comprising RNA sequencing data of total types of cancer, DNA copy digital data, variant annotation files, intron expression data, and clinical evaluation of colorectal cancer patients at home and abroad (http://gdac.broad institute website) were used in this study. Expression (raw counts and kilobase transcripts per million reads (FPKM)) data were normalized by quantile normalization. The CPTAC dataset used here contained the expression level of LSR protein in 111 LUAD tissues obtained from the Clinical Proteomic Tumor Analysis Consortium (https://cptac-data-portal.georgetown.edu/).

### 2.2. GO and KEGG Pathway Analyses

The database was used to classify target genes from RNA sequences for annotation, visualization, and comprehensive discovery (DAVID v6.8; https://david.ncifcrf.gov) based on Gene Ontology (GO) gene expression function annotation, pathway enrichment analysis, and Kyoto Encyclopedia of Genes and Genomes (KEGG) database. A cutoff value of *P* < 0.05 was used.

### 2.3. Cell Lines and Cell Culture

Human lung cancer cell lines H1299 and A549 were ordered from the American Type Culture Collection (ATCC) and cultured in DMEM with 10% FBS under a 37°C incubator containing 5% CO_2_.

### 2.4. RNA Extraction and qRT-PCR

Whole RNA was harvested by the TRIzol Kit (Omega, Norcross, GA, USA) and qualified by NanoDrop equipment (Thermo Fisher Scientific, Waltham, MA, USA). The cDNA Synthesis Kit (Takara, Otsu, Japan) was applied to synthesize complementary DNA (cDNA). Real-time PCR was conducted utilizing SYBR Green PCR Master Mix (Takara) in a StepOnePlus RT-PCR system (Thermo Fisher Scientific). The expression of all target genes was normalized to that of the internal gene GAPDH using the 2^-*ΔΔ*Ct^ method. The primers were as follows: LSR: 5′-TGACCGTGTCCAACCCCTA-3′, 5′-GGTCCCGGCAGAAAGACTT-3′; GAPDH: 5′-GGAGCGAGATCCCTCCAAAAT-3′, 5′-GGCTGTTGTCATACTTCTCATGG-3′.

### 2.5. siRNA Preparation and Transfection

The sequences of small interfering RNA (siRNA) targeting different human LSR were synthesized and ordered from GenePharma (Shanghai, China). Indicated cells were seeded into six-well plates and cultured for 24 hours before transfection. On the following day, all cells were transfected with indicated siRNAs using Lipofectamine 2000 (Invitrogen, Carlsbad, CA, USA) as the manual described. qRT-PCR was executed to determine the transfection efficiency. The siRNAs were as follows: si-LSR: 5′-GGACGACCTCTATGACCAA-3′; si-NC: 5′-UUCUCCGAACGUGUCACGUTT-3′.

### 2.6. CCK-8 Assay

A total of 2 × 10^3^ cells were seeded into 96-well plates. The CCK-8 detection kit (Tatsudo, Japan) was applied to detect cell proliferation. 10 *μ*l of CCK-8 solution was supplemented at 0, 1, 2, 3, and 4 days. A microtiter plate reader was used to measure the optical density at 450 nm. The cell survival rate was expressed by absorbance. A total of three repetitions were calculated under the same conditions to represent the results.

### 2.7. Transwell Migration and Invasion Assay

We prepared the cell suspension with a final standard of 5 × 10^4^ cells/ml. For the Transwell migration assay, 4 × 10^4^ cells in the 0.1 ml serum-free medium were transferred into the above chamber and DMEM with 10% FBS was added into the below chamber. All cells were incubated for 24 hours. All cells were collected and removed from the membrane, then stained with DAPI solution at room temperature for 10 minutes. For invasion assay, the upper chamber was coated with Matrigel before adding cells. All the derived data of cell migration and invasion was normalized to that of cell proliferation at 24 hours in case of the effects from cell proliferation.

### 2.8. Statistical Analysis

The Mann-Whitney *U* test, Student's *t*-test, and Fisher's exact test were conducted to assess the relationship between variables. The overall survival rate (OS) curve was drawn referring to the Kaplan-Meier method, and the logrank test was used to make a comparison. The Cox proportional hazard model was applied for univariate and multivariate analyses for further determining the predictive independent variables of OS. *P* ≤ 0.05 indicated a significant difference between or among indicated groups.

## 3. Results

### 3.1. LSR Was a Promising Oncogene in Lung Cancer

Through the bioinformatics analysis of TCGA dataset, we found that LSR might be a potential oncogene of lung cancer. Given TCGA dataset, we found that LSR expression in lung cancer tissues was greatly higher than that in normal lung tissues (Figure 1(a)). We got a similar result that LSR protein expression of 111 lung cancer patients' tissues in the CPTAC dataset was higher than that of normal tissues (Figure 1(b)). In conclusion, LSR was a potential gene for lung cancer.

### 3.2. High Expression of LSR in Lung Cancer Was Related to Metastasis Status, Grades, and Tumor Stages

Through clinicopathological analysis, we found that in LUAD, the increase of the LSR expression level was positively related to nodal metastasis status using TCGA database (Figure 1(c)). The increase of the LSR protein expression level was positively related to tumor grades using the CPTAC database (Figure 1(d)). Unfortunately, we could not analyze the correlation between LSR expression and nodal metastasis status in the CPTAC database and the correlation between LSR expression and tumor grades in TCGA database. Very interestingly, we found that the expression level of LSR in each stage of LUAD was higher than that in normal. However, the expression of LSR among different stages of LUAD was not observed to have a significant difference using both TCGA (Figure 1(e)) and CPTAC datasets (Figure 1(f)).

### 3.3. Increased Expression of LSR in Patients with Lung Cancer Exhibited an Association with Poor Survival

According to the expression of LSR in TCGA database, the patients were classified into 239 cases of high and 239 cases of low expressed LSR groups. We analyzed the correlation between survival time and LSR expression and found that the OS and DFS in patients with high LSR expression were reduced (Figures 2(a) and 2(b)). Besides, Kaplan-Meier analysis also revealed that high expression of LSR in NSCLC (Figures 2(c) and 2(d)) and LUAD (Figures 2(e) and 2(f)) was a factor of poor prognosis.

### 3.4. GO Term and KEGG Pathway Enrichment Analyses

We downloaded lung cancer-related data from TCGA and uploaded all DEGs to the online software DAVID to determine the overrepresented GO term and KEGG pathway. The data from GO analysis suggested that DEGs were primarily involved in the integrin-mediated signaling pathway, negative regulation of cell migration, cell migration, etc. (Figure 3(a)). KEGG functional analysis indicated that total DEGs were dominantly enriched in 10 KEGG metabolic pathways, including FoxO signaling pathway, ErbB signaling pathway, Epstein-Barr virus infection, apoptosis, NSCLC, endocytosis, focal adhesion, Fc gamma R-mediated phagocytosis, tight junction, and regulation of actin cytoskeleton (Figure 3(b)). These genes perhaps displayed a key role in cancer occurrence and development.

### 3.5. Knockdown of the LSR Gene Retarded Cell Proliferation, Migration, and Invasion of Lung Cancer

We further determined the effects of the LSR knockdown on lung cancer cell proliferation using the CCK-8 method. After transfection of si-LSR into lung cancer cell lines, LSR expression in A549 and H1299 cells was significantly decreased (Figure 4(a)). CCK-8 analysis data revealed that reduced expression of LSR dramatically hindered A549 and H1299 cell proliferation (Figure 4(b)).

In order to study the role of LSR in migration and invasion, A549 and H1299 cells were transfected with si-LSR as indicated. The data revealed that cell migration and invasion were decreased in a siRNA-transfected group after comparison with the control group (Figure 4(c)). In summary, LSR promoted cell proliferation, migration, and invasion of lung cancer cells.

## 4. Discussion

LSR, a type I single-pass transmembrane protein, is primarily expressed in the liver, intestine, and other tissues [14]. Upregulated LSR was demonstrated in various cancers, including colon, bladder, breast, endometrial, and ovarian cancers [15]. Numerous studies imply that LSR probably participates in the development of multiple cancers [16]. For instance, LSR is one of the most upregulated genes associated with metastasis progression *in vivo* [17]. Additionally, LSR induces invasion and migration of bladder cancer and aggressive breast cancer [14, 18]. In human colon cancer, the LSR expression level is revealed to be related to poor prognosis [19]. Recently, one study suggests that reduced LSR could promote cell migration, invasion, and proliferation of endometrial cancer cells [20]. Overexpressed LSR is currently considered a novel indicator of clinical prognosis and a potential therapeutic target in gastric cancer and colon cancer [21]. In this study, we evaluated the clinicopathological and oncogenic character of LSR in lung cancer and found that LSR mRNA and protein levels were upregulated in NSCLC and correlated to an advanced stage and shorter survival time of NSCLC. These results suggested that LSR is a potential biomarker for NSCLC.

Also, in this study, we performed a bioinformatics analysis of LSR. Very interestingly, we revealed that LSR was related to regulating the FoxO signaling pathway and ErbB signaling pathway. FoxO, a subfamily of the forkhead transcription factor, is believed to play an important role as a tumor suppressor in a variety of cancers [22]. FoxO is involved in the process of cell apoptosis, triggering the expression of a series of death receptor ligands such as TNF apoptotic ligand, Fas ligand, and bNIP3 [23]. FoxO interacts with some other important pathways like PI3K/AKT, AMPK, and RAS-MEK-ERK in tumorigenesis [24]. The ErbB signaling pathway includes the tyrosine kinase family-like EGFR and is associated with drug, chemotherapy, and radiation resistance in cancer. ErbB receptors, especially ErbB2 and EGFR, are overexpressed in many cancers such as non-small-cell lung cancer, ovarian cancer, and breast cancer. Moreover, EGFR binds to specific ligands to phosphorylate tyrosine residues which next initiate a variety of signal pathways such as the RAS-RAF-MEK-ERK pathway [25]. In summary, LSR may be involved in mediating the occurrence and development of lung cancer by regulating the FoxO signaling pathway and the ErbB signaling pathway.

Human cancer has hallmark characteristics, such as continued proliferation. The characteristic of continuous proliferation can be achieved by mutations in oncogenes and tumor suppressors that regulate cell growth [26]. Cancer cell migration is a plastic and adaptive process involving cytoskeleton dynamics, cell-extracellular matrix and cell-cell adhesion, and tissue remodeling [27]. Cancer cells use a variety of invasion and spread strategies, including collective and single-cell migration plans, to provide a basis for adapting to the microenvironment and treatment challenges [28]. Studying cell proliferation, migration, and invasion ability *in vitro* is a useful tool to assess the aggressiveness of solid cancers (including lung cancer) [29]. In *in vitro* functional experiment, we found that the proliferation ability of lung cancer cells was suppressed significantly after LSR downregulation. Besides, the metastasis ability of lung cancer cells was also significantly suppressed after the LSR knockdown. Furthermore, we verified that LSR promoted cell proliferation, migration, and invasion by upregulating its expression in lung cancer. In summary, we assessed the impacts of LSR expression on tumorigenesis and patient outcomes, hoping to provide a suitable direction for the discovery and treatment of lung cancer.

This study has some limitations. First, it is necessary to analyze the expression level of LSR in clinical samples. In future research, we will collect clinical samples and clinical parameters to explore the expression level and prognostic value of LSR. Second, it is necessary to further explore the function of LSR in lung cancer *in vivo*. We will explore the function of LSR in the lung cancer tumor-bearing mouse model. In addition, we will further explore the regulatory mechanisms of LSR and FoxO signaling and ErbB signaling pathways.

In summary, LSR was located on Ch.9q and was found to be an oncogene that is increased in lung cancer. The expression of LSR was related to tumor progression and poor prognostic status in lung cancer patients. Through bioinformatics analysis, it was found that LSR plays an important role in the progression of lung cancer. Functional experiments revealed that the knockdown LSR could impede lung cancer cell proliferation, migration, and invasion. Taken together, our data indicated that LSR was a prospective biomarker for prognosis and a target for lung cancer therapy.

## Figures and Tables

**Figure 1:** The clinical significance of LSR expression in lung cancer. (a) LSR expression in LUAD tissues and normal tissues in The Cancer Genome Atlas (TCGA) data. (b) LSR protein expression in LUAD tissues and normal tissues in the Clinical Proteomic Tumor Analysis Consortium (CPTAC) data. (c) LSR expression in LUAD based on the status of lymph node metastasis in TCGA data. (d) Expression of LSR protein in LUAD based on tumor malignancy in CPTAC data. (e) Expression of LSR in LUAD based on individual cancer stages in TCGA data. (f) Expression of LSR protein in LUAD based on cancer stages in CPTAC data.

**Figure 2:** The high expression level of LSR was significantly related to the reduction of OS and DFS in lung cancer. Kaplan-Meier OS (a) and DFS (b) curves of LUAD patients given LSR expression using TCGA dataset (*n* = 478). Kaplan-Meier analysis was performed on the OS (c) and DFS (d) curves of NSCLC patients with low or high LSR expression. Kaplan-Meier analysis was performed on the OS (e) and DFS (f) curves of LUAD patients with low or high LSR expression.

**Figure 3:** Knockdown of LSR participated in various signaling pathways in lung cancer cells. (a) The Gene Ontology term enrichment analysis of DEGs, significantly enriched in biological processes. (b) The KEGG pathway enrichment analysis of DEGs, mainly enriched in 9 pathways.

**Figure 4:** Knockdown of the LSR gene inhibited cell proliferation, migration, and invasion of lung cancer. (a) Reduced A549 and H1299 cell proliferation transfected with si-LSR. ^∗^*P* < 0.05. (b) CCK-8 assay analysis of cell proliferation in transfected A549 and H1299 cells. (c) Transwell assay analysis of the effect of si-LSR on cell migration and invasion abilities in A549 and H1299. ^∗^*P* < 0.05.

## Data Availability

The datasets used and/or analyzed during the current study are available from the corresponding author on reasonable request.
